The article "Serum Levels of lncRNA CCHE1 and TCF21 in Patients with Coronary Artery Disease and Their Clinical Significances" was published in 2021. Journal: Dis Markers.

# Serum Levels of lncRNA CCHE1 and TCF21 in Patients with Coronary Artery Disease and Their Clinical Significances

**DOI:** 10.1155/2021/8526144

**Published:** 2021-12-21

**Authors:** Miaomiao Liu, Ying Zhang, Xiantong Cao, Xue Wang

**Affiliations:** Department of Cardiovascular Surgery, First Affiliated Hospital of Xi'an Jiaotong University, Xi'an, China

## Abstract

**Objective:**

To detect serum level changes of CCHE1 and TCF21 in coronary artery disease (CAD) patients and to explore their clinical significances. *Patients and Methods*. A total of 150 CAD patients were divided into the mild lesion group (*n* = 52), moderate lesion group (*n* = 48), and severe lesion group (*n* = 50), respectively, according to the Gensini score. In addition, they were divided into single vessel lesion (*n* = 42), two vessel lesions (*n* = 49), and three vessel lesions group (*n* = 59), respectively. Serum levels of CCHE1 and TCF21 in CAD patients were detected by quantitative real-time polymerase chain reaction (qRT-PCR). Spearman's rank correlation was conducted to assess the relationship between levels of CCHE1 and TCF21 and severity and numbers of vessel lesions in CAD. Pearson's correlation test was used for analyzing the correlation between CCHE1 and TCF21 levels. A multivariable logistic regression test was performed to evaluate the influences of CCHE1 and TCF21 levels on CAD severity and the occurrence of cardiovascular events within 3 years of follow-up.

**Results:**

Significant differences in incidences of diabetes and hypertension were identified in CAD patients divided according to CAD severity. In addition, significant differences in incidences of drinking, diabetes, and hypertension were identified in CAD patients divided according to numbers of vessel lesions. The serum level of CCHE1 was positively related to CAD severity and numbers of vessel lesions, while TCF21 displayed a negative relationship. During the 3-year follow-up, the incidence of cardiovascular events was 39.3% (59/150). CAD severity, numbers of vessel lesions, and serum levels of CCHE1 and TCF21 were independent factors influencing the occurrence of cardiovascular events in CAD patients.

**Conclusions:**

The increased serum level of CCHE1 and decreased TCF21 level are closely related to CAD severity, which are able to influence the prognosis in CAD patients.

## 1. Introduction

Coronary artery disease (CAD) is one of the major reasons for global death [1]. CAD is mainly caused by atherosclerosis [2]. Phenotypes of vascular smooth muscle cells (VSMCs) are changed following injuries, and they migrate to intima and aggregate ECM. VSMCs are of significance in the development of atherosclerosis [3].

The article "Serum Levels of lncRNA CCHE1 and TCF21 in Patients with Coronary Artery Disease and Their Clinical Significances" was published in 2021. Journal: Dis Markers.

Long non-coding RNAs (lncRNAs) contain more than 200 nucleotides in length, and they are unable to encode proteins [4]. Abnormally expressed lncRNAs have been detected in the heart or circulating system of myocardial infarction (MI) patients [5, 6]. A latest study has uncovered that lncRNA LIPCAR is capable of monitoring heart failure at post-MI, serving as a promising biomarker [7]. Further, MIAT controls advanced atherosclerotic lesion formation and plaque destabilization [8]. The SNHG1-driven self-reinforcing regulatory network promoted cardiac regeneration and repair after myocardial infarction [9]. lncRNA CCHE1 (cervical carcinoma high expressed 1) has been recently discovered [10]. Microarray analysis showed upregulated CCHE1 in breast cancer profiling, suggesting that CCHE1 may have a certain impact on breast cancer progression [11, 12]. The correlation between CCHE1 and CAD, however, is rarely reported.

TCF21 locates on 6q23-q24, which was discovered in the research on the location of chromosomal heterozygosity in 2006 by Smith et al. [13]. TCF21 is a metastasis-suppressor gene. It is reported that TCF21 is extensively expressed in stromal cells or derived cells during the development of cardiovascular system, urogenital system, and respiratory system [14]. It largely affects cell growth and differentiation. A previous study has proposed that LINC00163 alleviates lung cancer progression by upregulating TCF21 [15]. In this paper, we mainly explored the clinical significances of CCHE1 and TCF21 in CAD patients. Our findings can provide novel ideas in clinical treatment of CAD.

## 2. Patients and Methods

### 2.1. Baseline Characteristics

A total of 150 patients admitted in our hospital from June 2017 to May 2019 because of chest tightness, chest pain, or acute MI were enrolled. All patients underwent coronary angiography and treated according to the “2012 ACCF/AHA Focused Update of the Guideline for the Management of Patients with Unstable Angina/non-ST-Elevation Myocardial Infarction” [16]. Gensini score was graded depending on the stenosis and the locations of vessel narrowing (1 grade: stenosis < 25%, 2 grades: 26%-50% stenosis, 4 grades: 51-75% stenosis, 8 grades: 76%-90%, 16 grades: 90%-98%, and 32 grades: complete stenosis) [17]. Then, the corresponding coefficients were determined by the location of different narrowing branches of coronary artery (left coronary artery: ×5, proximal LAD: ×2.5, mid-LAD: ×1.5, and distal LAD: ×1). We divided CAD patients into the mild lesion group (1.0-26.1 grades, *n* = 52), the moderate lesion group (26.2-51.4 grades, *n* = 48), and the severe lesion group (≥51.5 grades, *n* = 50) according to the Gensini score. In addition, patients were classified by the number of vessel lesions to the single-vessel lesion group: ≥50% of stenosis of any single vessel in LAD, left circumflex, and right coronary artery; the two-vessel lesion group: ≥50% of stenosis of any two vessels in LAD, left circumflex and right coronary artery; three vessel lesions group: stenosis in LAD, left circumflex and right coronary artery, or lesions in left main coronary artery combined with the right coronary artery. Patients with malignant tumors, liver or kidney insufficiency, acute/chronic infection, pregnant or lactating women, or those unwilling to participate in were excluded. The study was reviewed and approved by the Ethics Committee of First Affiliated Hospital of Xi'an Jiaotong University. All patients signed the informed consent.

The article "Serum Levels of lncRNA CCHE1 and TCF21 in Patients with Coronary Artery Disease and Their Clinical Significances" was published in 2021. Journal: Dis Markers.

### 2.2. Laboratory Examinations

Serum levels of TC (total cholesterol), TG (triglyceride), LDL-C (low-density lipoprotein cholesterol), and HDL-C (high-density lipoprotein cholesterol) were determined using the automatic biochemical instrument. Hcy (homocysteine) and CRP (C-reactive protein) were detected by enzyme-linked immunosorbent assay (ELISA) (R&D Systems, Minneapolis, MN, USA). LVEF (left ventricular ejection fraction) was recorded by echocardiography.

### 2.3. Quantitative Real-Time Polymerase Chain Reaction (qRT-PCR)

Serum RNA was isolated using TRIzol and quantified by NanoDrop 2000 (Thermo Fisher Scientific, Waltham, MA, USA). RNA was reversely transcribed to complementary deoxyribose nucleic acid (cDNA) with the PrimeScript™ RT Master Mix and amplified by TBGreen® Premix Ex Taq™ II (TaKaRa, Tokyo, Japan). Thermal cycle reactions were as follows: 30 s at 95°C and 40 cycles for 5 s at 95°C and 30 s at 60°C. Primer sequences were as follows: CCHE1—5′-AAGGTCCCAGGATACTCGC-3′ (forward) and 5′-GTGTCGTGGACTGGCAAAAT-3′ (reverse); TCF21—5′-CCAGCTACATCGCCCACTTG-3′ (forward) and 5′-CTTTCAGGTCACTCTCGGGTTTC-3′ (reverse); and GAPDH—5′-ACCACAGTCCATGCCATCAC-3′ (forward) and 5′-TCCACCACCCTGTTGCTGTA-3′ (reverse).

### 2.4. Follow-Up

Patients were followed up for three years by review, telephone, or e-mail. Cardiovascular events were recorded, including angina pectoris, MI, arrhythmia, sudden cardiac death, and stroke.

### 2.5. Statistical Analyses

Data were processed by SPSS 20.0. Measurement data were expressed as the mean ± SD and compared using a *t*-test or variance analysis. Counting data were expressed as composition ratio or rate (%) and compared by a chi-square test. Spearman's rank correlation was conducted to assess the relationship between levels of CCHE1 and TCF21 and severity and numbers of vessel lesions in CAD. Pearson's correlation test was used for analyzing the correlation between CCHE1 and TCF21 levels. A multivariable logistic regression test was performed to analyze the influences of CCHE1 and TCF21 levels on CAD severity and the occurrence of cardiovascular events within 3 years of follow-up. *p* < 0.05 was statistically significant.

The article "Serum Levels of lncRNA CCHE1 and TCF21 in Patients with Coronary Artery Disease and Their Clinical Significances" was published in 2021. Journal: Dis Markers.

## 3. Results

### 3.1. Clinical Data of CAD Patients

Significant differences in incidences of diabetes and hypertension were identified in CAD patients in the mild lesion group (*n* = 52), the moderate lesion group (*n* = 48), and the severe lesion group (*n* = 50) divided according to the Gensini score. Besides, significant differences in incidences of drinking, diabetes and hypertension were identified in CAD patients in the single-vessel lesion (*n* = 42), two-vessel lesion (*n* = 49), and three-vessel lesion groups (*n* = 59) (Tables 1 and 2). It is indicated that diabetes and hypertension could affect CAD severity, while diabetes, hypertension, and drinking could affect numbers of vessel lesions.

### 3.2. Serum Levels of CCHE1 and TCF21 in CAD Patients with Different Severities

Serum levels of CCHE1 and TCF21 in CAD patients with different severities were detected by qRT-PCR. CCHE1 level increased with the aggravation of CAD, manifesting as the lowest level in the mild lesion group and the highest level in the severe lesion group (Figure 1(a)). On the contrary, TCF21 level decreased with the severity of CAD (Figure 1(b)).

### 3.3. Serum Levels of CCHE1 and TCF21 in CAD Patients with Different Numbers of Vessel Lesions

We thereafter detected CCHE1 and TCF21 levels in CAD patients classified by numbers of vessel lesions. The lowest level of CCHE1 was detected in the single-vessel lesion group, and the highest level was detected in the three-vessel lesion group (Figure 2(a)). TCF21 level gradually decreased with the increased numbers of vessel lesions (Figure 2(b)).

### 3.4. Relationship between Levels of CCHE1 and TCF21 and Severity and Numbers of Vessel Lesions in CAD

Spearman's rank correlation results uncovered that CCHE1 level was positively correlated to CAD severity and numbers of vessel lesions (*r* = 0.388 and 0.671, respectively, *p* < 0.05), whereas TCF21 displayed a negative correlation to them (*r* = −0.523 and -0.397, respectively, *p* < 0.05) (Table 3). It is further supported that CCHE1 and TCF21 were involved in the progression of CAD. In particular, CCHE1 aggravated CAD and TCF21 exerted a protective role.

### 3.5. Negative Interaction between CCHE1 and TCF21 in CAD Patients

Pearson's correlation test was conducted to elucidate the potential interaction between CCHE1 and TCF21 in CAD patients. As data revealed, the serum level of CCHE1 was negatively correlated to TCF21 (*r* = −0.5099, *p* < 0.001) (Figure 3).

The article "Serum Levels of lncRNA CCHE1 and TCF21 in Patients with Coronary Artery Disease and Their Clinical Significances" was published in 2021. Journal: Dis Markers.

### 3.6. Influences of CCHE1 and TCF21 Levels on Cardiovascular Events in CAD Patients

During the 3-year follow-up, the incidence of cardiovascular events was 39.3% (59/150). Variables with statistical significances in Tables 1 and 2 were assigned as independent ones as follows: diabetes (yes = 1, no = 0); hypertension (yes = 1, no = 0); drinking (yes = 1, no = 0); CAD severity (mild lesion = 1, moderate and severe lesion = 2); and numbers of vessel lesions (single vessel = 1, multiple vessels = 2). Subsequently, CAD patients were divided into two groups according to the cut-off values of mRNA levels of CCHE1 and TCF21 (high level = 1, low level = 0). The occurrence of cardiovascular events during the follow-up of CAD patients was assigned as the dependent variable (yes = 1, no = 0). A multivariable logistic regression test demonstrated that severe CAD, multiple vessel lesions, and high level of CCHE1 were independent risk factors, while the high level of TCF21 was a protective factor influencing the occurrence of cardiovascular events in CAD patients (Table 4).

## 4. Discussion

With the completion of the gene sequencing program and the development of molecular biology, it is found that protein-encoding mRNAs only account for 2% of the human genome. More than 95% of the transcribed sequences in the genome are noncoding RNAs [18]. These noncoding RNAs, which were initially regarded as nonfunctional, are involved in various life activities. As a family member of noncoding RNAs, lncRNAs are 200 bp long. They exert diverse functions as signal molecules, decoy molecules, and scaffold molecules. lncRNAs are involved in genetic, transcriptional, and posttranscriptional regulations [19].

lncRNAs have been identified to have a relation to vascular diseases. It is reported that lncRNA ANRIL is highly expressed in the blood of atherosclerosis patients, and the high level of ANRIL enhances the risk of MI [20, 21]. Circulating system lncRNAs are promising biomarkers for diagnosing ischemic heart diseases. For example, lncRNA LIPCAR is linked to the progression of heart failure, which serves as a molecular indicator for myocardial remodeling [22]. Upregulated plasma lncRNA CoroMarker is highly specific and sensitive for diagnosing CAD [23]. Through regulating VSMC phenotypes, lncRNAs regulate atherosclerosis development by mediating adipogenesis and lipid deposition [24].

CCHE1 is upregulated in cervical cancer specimens and correlated to tumor size, tumor staging and overall survival in cervical cancer patients. It is considered a potential therapeutic target and prognostic biomarker for cervical cancer [25]. Meanwhile, CCHE1 is highly expressed in non-small-cell lung carcinoma, which drives malignant phenotypes *via* the ERK/MAPK signaling [26]. Overexpression of CCHE1 triggers proliferative rate and inhibits apoptosis of gastric cancer cells [27]. Our findings detected an increased serum level of CCHE1 in CAD patients, and its level was elevated with the aggravation of CAD. The high level of CCHE1 enhanced the risk of cardiovascular events in CAD patients.

The article "Serum Levels of lncRNA CCHE1 and TCF21 in Patients with Coronary Artery Disease and Their Clinical Significances" was published in 2021. Journal: Dis Markers.

TCF21, also known as POD-1, belongs to the bHLH family. It is expressed in the mesenchymal cells of the lung, kidney, and intestine; cardiac interstitial cells [28]; and glomerular epithelial cells [29]. TCF21 is of significance in driving EMT [30–32]. Cao et al. [31] detected urine samples in 50 bladder cancer patients, 50 renal cancer patients, and 50 prostate cancer patients. They proposed that combined detection of TCF21 level and PCDH17 methylation is conductive to diagnose urinary system tumors. Ye et al. [33] showed that abnormal methylation of TCF12 is associated with the poor prognosis in clear cell renal cell carcinoma. TCF21 is also an independent factor influencing the progression of CAD [34, 35]. Consistently, we found that the serum level of TCF21 decreased in CAD patients. TCF21 exerted a protective role in CAD severity and numbers of vessel lesions. A negative correlation was identified between serum levels of CCHE1 and TCF21. We believed that enhanced level of CCHE1 and downregulated TCF21 predict the deterioration of CAD. In summary, we uncover the relationship between CCHE1 and TCF21 in CAD; however, the lack of *in vivo* and *in vitro* assay is the shortage of this research.

## 5. Conclusion

Increased serum level of CCHE1 and decreased TCF21 level are closely related to CAD severity, which are able to influence the prognosis in CAD patients.

## Figures and Tables

**Figure 1:** Serum levels of CCHE1 and TCF21 in CAD patients with different severities. Serum levels of CCHE1 (a) and TCF21 (b) in CAD patients of the mild lesion, moderate lesion, and severe lesion groups.

**Figure 2:** Serum levels of CCHE1 and TCF21 in CAD patients with different numbers of vessel lesions. Serum levels of CCHE1 (a) and TCF21 (b) in CAD patients of the single-vessel lesion, two-vessel lesion, and three-vessel lesion groups.

**Figure 3:** A negative correlation between serum levels of CCHE1 and TCF21 in CAD patients (*r* = −0.5099, *p* < 0.001).

**Table 1:** Clinical data of CAD patients with different severities.

Variable	Mild lesion (*n* = 52)	Moderate lesion (*n* = 48)	Severe lesion (*n* = 50)	*p*
Male/female	25/27	24/24	27/23	0.831
Age	56.23 ± 7.85	54.91 ± 6.08	55.21 ± 5.45	0.159
BMI (kg/m^2^)	24.73 ± 3.11	23.01 ± 3.65	23.83 ± 3.94	0.073
Smoking	20 (38.46%)	17 (35.42%)	23 (46%)	0.543
Drinking	12 (23.08%)	14 (29.17%)	15 (30%)	0.693
TC (mmol/L)	4.89 ± 1.07	4.08 ± 1.33	4.36 ± 1.54	0.615
TG (mmol/L)	1.64 ± 0.46	1.73 ± 0.55	1.74 ± 0.54	0.368
LDL-C (mmol/L)	1.44 ± 0.62	1.38 ± 0.56	1.43 ± 0.71	0.741
HDL-C (mmol/L)	2.56 ± 1.72	2.65 ± 1.48	2.71 ± 1.82	0.587
Hcy (mmol/L)	14.46 ± 2.88	15.84 ± 3.06	15.38 ± 2.89	0.087
CRP (mg/L)	12.27 ± 5.23	13.61 ± 5.66	13.84 ± 5.68	0.103
LVEF (%)	64.13 ± 10.22	62.33 ± 9.36	60.87 ± 8.91	0.067
Diabetes (%)	5 (9.62%)	4 (8.33%)	13 (26%)	0.021
Hypertension (%)	4 (7.69%)	7 (14.58%)	18 (16%)	0.001

BMI: body mass index; TC: total cholesterol; TG: triglyceride; LDL-C: low-density lipoprotein cholesterol; HDL-C: high-density lipoprotein cholesterol; Hcy: homocysteine; CRP: C-reactive protein; LVEF: left ventricular ejection fraction.

The article "Serum Levels of lncRNA CCHE1 and TCF21 in Patients with Coronary Artery Disease and Their Clinical Significances" was published in 2021. Journal: Dis Markers.

**Table 2:** Clinical data of CAD patients with different numbers of vessel lesions.

Variable	Single vessel (*n* = 42)	Two vessels (*n* = 49)	Three vessels (*n* = 59)	*p*
Male/female	23/19	22/27	31/28	0.601
Age	57.27 ± 6.95	55.68 ± 5.18	57.11 ± 6.13	0.338
BMI (kg/m^2^)	22.13 ± 4.03	23.32 ± 4.53	23.12 ± 3.83	0.275
Smoking	17 (40.48%)	19 (38.78%)	24 (40.68%)	0.977
Drinking	6 (14.29%)	10 (20.41%)	25 (42.37%)	0.003
TC (mmol/L)	4.11 ± 2.37	4.41 ± 2.54	4.26 ± 2.05	0.652
TG (mmol/L)	1.77 ± 0.73	1.86 ± 0.71	1.92 ± 0.83	0.076
LDL-C (mmol/L)	1.37 ± 0.51	1.48 ± 0.56	1.43 ± 0.71	0.198
HDL-C (mmol/L)	2.56 ± 1.72	2.73 ± 1.98	2.82 ± 2.13	0.227
Hcy (mmol/L)	13.86 ± 3.18	14.21 ± 3.22	14.88 ± 3.89	0.088
CRP (mg/L)	12.57 ± 5.95	13.61 ± 5.99	14.11 ± 6.18	0.367
LVEF (%)	65.03 ± 11.73	63.13 ± 10.43	61.07 ± 9.32	0.216
Diabetes (%)	2 (4.76%)	6 (12.24%)	14 (23.73%)	0.025
Hypertension (%)	4 (9.52%)	6 (12.24%)	19 (32.2%)	0.005

BMI: body mass index; TC: total cholesterol; TG: triglyceride; LDL-C: low-density lipoprotein cholesterol; HDL-C: high-density lipoprotein cholesterol; Hcy: homocysteine; CRP: C-reactive protein; LVEF: left ventricular ejection fraction.

**Table 3:** Relationship between levels of CCHE1 and TCF21 and severity and numbers of vessel lesions in CAD.

	CCHE1		TCF21	
	*r*	*p*	*r*	*p*
Severity of CAD	0.388	0.041	-0.523	0.022
Numbers of vessel lesions	0.671	0.003	-0.397	<0.001

**Table 4:** Multivariable logistic analysis on potential factors influencing the occurrence of cardiovascular events in CAD patients.

Variable	OR	95% CI	*p*
Diabetes	1.733	0.614-5.332	0.142
Hypertension	0.892	0.561-2.313	0.668
Drinking	0.873	0.446-2.985	0.079
Severity of CAD	1.681	1.281-3.452	0.035
Number of vessel lesions	1.546	1.332-2.775	<0.001
CCHE1	2.387	1.654-5.872	<0.001
TCF21	0.584	0.287-1.664	0.007

The article "Serum Levels of lncRNA CCHE1 and TCF21 in Patients with Coronary Artery Disease and Their Clinical Significances" was published in 2021. Journal: Dis Markers.

## Data Availability

The datasets used and analyzed during the current study are available from the corresponding author on reasonable request.
